This article has been retracted.

# Comparison of acupuncture and other drugs for chronic constipation: A network meta-analysis

**DOI:** 10.1371/journal.pone.0196128

**Published:** 2018-04-25

**Authors:** Lingping Zhu, Yunhui Ma, Xiaoyan Deng

**Affiliations:** 1 General Practice Department of Shenzhen Longhua District Central Hospital, Shenzhen, Guangdong Province, China; 2 General Practice Department of Zhongshan Hospital of Fudan University, Shanghai City, China; 3 Endocrinology Department of Shenzhen Longhua District Central Hospital, Shenzhen, Guangdong Province, China; University Hospital Llandough, UNITED KINGDOM

## Abstract

The objective of this study was to compare the efficacy and side effects of acupuncture, sham acupuncture and drugs in the treatment of chronic constipation. Randomized controlled trials (RCTs) assessing the effects of acupuncture and drugs for chronic constipation were comprehensively retrieved from electronic databases (such as PubMed, Cochrane Library, Embase, CNKI, Wanfang Database, VIP Database and CBM) up to December 2017. Additional references were obtained from review articles. With quality evaluations and data extraction, a network meta-analysis (NMA) was performed using a random-effects model under a frequentist framework. A total of 40 studies (n = 11032) were included: 39 were high-quality studies and 1 was a low-quality study. NMA showed that (1) acupuncture improved the symptoms of chronic constipation more effectively than drugs; (2) the ranking of treatments in terms of efficacy in diarrhoea-predominant irritable bowel syndrome was acupuncture, polyethylene glycol, lactulose, linaclotide, lubiprostone, bisacodyl, prucalopride, sham acupuncture, tegaserod, and placebo; (3) the ranking of side effects were as follows: lactulose, lubiprostone, bisacodyl, polyethylene glycol, prucalopride, linaclotide, placebo and tegaserod; and (4) the most commonly used acupuncture point for chronic constipation was ST25. Acupuncture is more effective than drugs in improving chronic constipation and has the least side effects. In the future, large-scale randomized controlled trials are needed to prove this. Sham acupuncture may have curative effects that are greater than the placebo effect. In the future, it is necessary to perform high-quality studies to support this finding. Polyethylene glycol also has acceptable curative effects with fewer side effects than other drugs.

## Introduction

Chronic constipation is a very common condition that can affect a patient's quality of life. Symptoms of constipation include decreased intestinal motility, stool consolidation, frequent forced bowel movements, bloating, urge to defecate, and abdominal discomfort. [1] The proportion of people affected by chronic constipation varies widely, accounting for 0.7%-29.6% of children and 2%-35% of adults in Europe [2]. The prevalence of chronic constipation in North America is estimated to be 2% to 27% due to differences in the diagnostic criteria. [3] Consultations for constipation account for 2.5 million visits per year in the United States [4]. Constipation is associated with a large financial burden to patients and the country; one study showed that the cost for each patient during the diagnostic process of constipation was approximately 2757 dollars [5]. Studies have shown that the causes of constipation include many factors such as diet, drugs, metabolic or neurological diseases, psychosocial factors, and disorders of colonic motility and defecation. [6]

The methods of treating chronic constipation currently include drugs and acupuncture. Common drugs include lactulose, polyethylene glycol, linaclotide, lubiprostone, bisacodyl, prucalopride, tegaserod, etc. But most of drugs have some side effects which couldn’t be tolerated by patients, complementary or alternative treating methods with less side effect are needed in our practice. An increasing number of studies have shown that acupuncture may have certain effects on chronic constipation. However, there have been no studies comparing acupuncture and commonly used oral drugs. The comparison between drugs and acupuncture will bring us a clear understanding of those interventions. Furthermore, various acupoints have been targeted to treat chronic constipation. Therefore, this study was designed to solve these unanswered questions.

This study was a systematic review of the literature and collected data from published randomized controlled trials (RCTs) of acupuncture and common oral drugs in the treatment of chronic constipation up to December 2017. This study aimed to answer the following questions: (1) what are the curative effects and side effects of acupuncture and drugs to improve chronic constipation?; (2) what is the curative effect of sham acupuncture as a placebo?; and (3) what are the acupoints to cure constipation?

## Materials and method

We followed the protocols based on the preferred reporting item[7,8] of the PRISMA(Preferred Reporting Items for Systematic Reviews and Meta Analyses) statement.

### Research methods

We searched PubMed, the Cochrane Library, Embase and 4 Chinese databases [China National Knowledge Infrastructure (CNKI), Wanfang Database, VIP Database and Chinese Biomedical Database (CBM)] to conduct a comprehensive database retrieval, the retrieval time is from the time of database building to February 2018. The following search keywords were used: (lactulose, polyethylene glycol, linaclotide, lubiprostone, bisacodyl, prucalopride, tegaserod), (randomized controlled trials or clinical trials), and (IBS-D) (see appendix). In addition, manual searches of the reference lists of review articles and meta-analyses were conducted. No language restrictions were set.

### Inclusion and exclusion criteria

We included RCT and publications that met the following eligibility criteria: (i) clinical trials of adult patients; (ii) clinical trials of single drugs; (iii) clinical trials with treatment duration greater than two weeks; (iv) publications that were not comments or commentaries; and (v) studies that excluded pregnant or lactating women, patients with peptic ulcers, rectal disease, or liver or other systemic disease, and patients with previous history of gastroduodenal surgery, neurologic diseases or neurologic surgery.

### Research options

Articles were independently screened by two researchers. Initially, the NoteExpress Software (Beijing Aegean Sea Music Technology Co., Ltd.) was used to delete duplicate records. The remaining summaries and full texts were reviewed based on the above inclusion and exclusion criteria, and disagreements were resolved through discussion.

### Data extraction and quality assessment

Two reviewers (Lingping Zhu and Xiaoyan Deng) independently extracted the relevant information from each eligible study using a pre-prepared data extraction sheet. Data collected included the location and study design of the trials, clinical characteristics of the patients, number of patients, patient age, diagnostic methods, treatment duration, outcome data, and side effects. The quality of the included studies was assessed using the Jadad Scale, which is based on the following three factors: randomized (2 points), double-blinded (2 points) and withdrawals and drop-outs (1 point) [9]. A Jadad score of 3 or higher was considered high quality. Disagreements were resolved by discussion.

The primary outcome was the proportion of patients with improvement in chronic constipation. Secondary outcomes were side effects and common acupuncture points. Common side effects included constipation and rash.

### Data synthesis and analysis

The assessments of acupuncture and drug efficacy were based on a combination of data extracted from the included trials. Direct and indirect comparisons were performed for the overall effect of acupuncture and medications. In thisNMA, we used a random-effects model in a Bayesian framework. The odds ratio (OR) and 95% confidence interval (CI) were used to analyse the effects of acupuncture and drugs on the efficacy of diarrhoea-predominant irritable bowel syndrome. CIs with OR> 1.0 indicated statistically significant, and CIs not containing 1.0 were considered statistically significant. All analyses were conducted using the GeMTC package generated by R software [10, 11].

Node-splitting models were used to assess the consistency of theNMA to test whether the results of the direct and indirect comparisons were consistent within the treatment cycle [12]. However, In the absence of direct or indirect comparison results, the node-splitting model could not be executed. Therefore, we used statistic analysis to quantify the degree of heterogeneity using I2 calculations. I2 > 50% was considered heterogeneous. To verify the robustness of the results, sensitivity analyses were performed in each study and recalculating the overall effect to see the individual effect of each factor.

A mesh diagram, contribution graphs, and publication bias tests were performed using STATA 14.0 software (Stata Corporation, College Station, TX, USA).

## Results

### 1. Characteristics of the included studies

A total of 1516 articles were obtained from the literature search. After reviewing the literature, 36 duplicates were deleted. After reviewing the inclusion criteria, 1438 articles were excluded. Finally, a total of 40 trials were identified (Fig 1) and are listed in S1 Table [13–51].

**Fig 1:** Flow diagram.

A total of 11032 patients with chronic constipation were enrolled across all studies. The studies investigated a total of 10 treatment modalities including A: prucalopride; B: tegaserod; C: lubiprostone; D linaclotide E: bisacodyl; F: PEG; G: lactulose; H: acupuncture; I: sham acupuncture; and J: placebo (sucrose, etc.). There were 12 articles from China, 11 articles from the United States, 7 articles from multiple countries, 4 articles from the UK, and 1 article each from France, Italy, Belgium, Germany, the Netherlands and Japan. The overall Jadad score for study quality ranged from 3–7. (Details in S1 Table)

### 2. Routine paired meta-analysis

Compared with placebo, acupuncture significantly improved the symptoms of chronic constipation (OR: 9.4, 95% CI: 3.6–9.7) (Fig 2). Polyethylene glycol, lactulose, and linaclotide also improved the symptoms of chronic constipation compared to placebo (OR: 6.5, 95% CI: 3.8–12.0; OR: 4.4, 95% CI: 2.0–9.7; and OR: 3.8, 95% CI: 2.4–6.4, respectively) (Fig 2). Compared with placebo, lubiprostone, bisacodyl, and prucalopride also improved the symptoms of chronic constipation (OR: 3.7, 95% CI: 2.1–6.6; OR: 3.4, 95% CI: 1.5–7.2; and OR: 2.7, 95% CI: 2.0–3.8, respectively) (Fig 2). Sham acupuncture also improved the symptoms of chronic constipation compared to placebo (OR: 3.1, 95% CI: 1.1–9.3). The effect of tegaserod was non-significant to that of placebo (OR: 1.7, 95% CI: 0.90–3.1, I2 = 0.0%) When acupuncture and oral medications were compared, the curative effect of oral medications was worse than that of acupuncture (for more details, see Fig 2). The I^2^ for polyethylene glycol, lactulose, linaclotide, lubiprostone, Bisacodyl and prucalopride compared with placebo are respectively 73.7%, 0%, 51.7%, 69.1%, 0% and 64.3%.

**Fig 2:** Forest plot of conventional meta-analysis for acupuncture and drugs to constipation. A:Prucalopride; B:Tegaserod; C:Lubiprostone; D:linaclotide; E:Bisacodyl; F:Polyethylene Glycol; G:lactulose; H:acupuncture+electroacupuncture; I:sham acupuncture; J:Placebo.

### 2. The cumulative probability ranking

By cumulative probability ranking, patients with chronic constipation were sorted by those receiving needle acupuncture, polyethylene glycol, lactulose, linaclotide, lubiprostone, bisacodyl, prucalopride, sham acupuncture, tegaserod, and placebo. Given that the probability distributions of linaclotide, lubiprostone, and bisacodyl were similar, we used the probability of the highest ranking. It was found that the efficacy of acupuncture was much higher than that of drugs (P = 0.75) and the efficacy of polyethylene glycol was higher (P = 0.50) than other drugs, including lactulose (P = 0.28), linaclotide (P = 0.20), lubiprostone (P = 0.23), bisacodyl (P = 0.16), prucalopride (P = 0.32), tegaserod (P = 0.70), and placebo (P = 0.93) (Fig 3 and S2 Table).

**Fig 3:** The cumulative probability ranking plot of treatment effect of acupuncture and other drugs on chronic constipation.

Twenty-two out of the 40 studies provided data regarding side effects (S1 Table). One study on acupuncture reported side effect data, while the other studies of acupuncture reported no side effects of acupuncture or sham acupuncture. The NMA cannot analyse isolated data so the side effects for acupuncture or sham acupuncture were not included in the final analysis. Twenty-one studies reported data on side effects of the remaining eight treatments (see S1 Table). Acupuncture had the fewest side effects, as there are not many known side effects, followed by mild side effects of tegaserod (P = 0.51) and linaclotide (P = 0.47). There were more side effects from lactulose (P = 0.55) and lubiprostone (P = 0.49) than other drugs. The side effects of the drugs are listed in Fig 4 and S3 Table.

**Fig 4:** The cumulative probability ranking plot of side effect of drugs on Chronic Constipation.

### 3. Network diagrams

We compared all of the included studies and drew network diagrams with the studies incorporated into quality-based displays on a network map. (Fig 5).

**Fig 5:** The network plot of all treatment methods, color means the mean quality of included studies, yellow means the low quality studies, green means the high quality studies.

### 4. Acupuncture preference points

Regarding the different acupuncture points selected for each study, we identified the most commonly used acupoints, including ST-25; the use of ST25 acupoints were counted 12 times compared to other acupoints which were 4 times at most (Table 1).

**Table 1:** Frequencies for all acupoints treating constipation.

Acupoints	Frequencies
ST25	12
ST37	4
SP6	2
SP14	2
BL24	1
BL26	1
ST28	1
CV4	1
ST36	1
CV6	1

### 5. Brooks-Gelman-Rubin diagnostic plot, density plot, node-splitting plot and cumulative contribution plot

By performing 20,000 convergence iterations, we obtained a Brooks-Gelman-Rubin diagnostic plot, and the track density map was acceptable; based on the node-splitting model, we found all studies in the region beneath the 4th line. We also obtained a cumulative contribution map from the STATA software (S1, S2, S3, and S4 Figs).

### 6. Heterogeneity

Using heterogeneity analysis, we found that polyethylene glycol, linaclotide, lubiprostone, and prucalopride had significant heterogeneity; based on the sensitivity analysis, we corrected the OR for polyethylene glycol (OR: 3.92, 95% CI: 2.70–5.71, I2 = 37%), linaclotide (OR: 3.11, 95% CI: 2.33–4.16, I2 = 0.0%), lubiprostone (OR: 2.80, 95% CI: 1.93–4.05, I2 = 16%), and prucalopride (OR: 2.78, 95% CI: 2.34–3.29, I2 = 48%). No large directional change occurred even after corrections (S5 and S6 Figs).

### 7. Publication bias

Using the funnel plot, all included studies were compared on a pairwise basis, and all studies were found to be essentially symmetrical, indicating a small publication bias (Fig 6).

**Fig 6:** The funnel plot of all included studies. PRU:Prucalopride; TEG:Tegaserod; LUB:Lubiprostone; LIN:linaclotide; BIS:Bisacodyl; PEG:Polyethylene Glycol; LAC:lactulose; ACU:acupuncture+electroacupuncture; SHAM ACU:sham acupuncture.

## Discussion

By including more than 40 articles for network meta-analysis(NMA), acupuncture was found to be more effective than drugs in treating chronic constipation with nearly no side effects. The mechanism of action of acupuncture for the treatment of chronic constipation remains unclear, but previous studies have also shown its possible role in the treatment of chronic constipation. An important cause of chronic constipation is the decreased motility of the colon, resulting in a decreased urge to defecate, bloating, and abdominal pain or discomfort. [51] Existing studies indicate that acupuncture at heterotopic acupoints facilitates distal colonic motor ability by activating M3 receptors and somatic afferent C-fibres in normal, constipated, or diarrhoeic rats. Acupuncture can also increase distal colonic motility in normal and abnormal mice with a possible role of M3 receptors [52]. Previous studies have suggested that the ST36 acupoint can change the motor function of the colon. [53]

However, a previous meta-analysis showed no significant curative benefits of acupuncture compared with sham acupuncture in the treatment of chronic constipation. Only some studies from China have shown that acupuncture is superior to drugs. [54] A previous study from China showed that acupuncture and sham acupuncture had similar effects on functional constipation, but moxibustion was used with ST23 and ST27 acupoints in this study. Moreover, this study was based on a small sample size [55], and therefore, we are unable to ensure the accuracy of these findings. In addition, the curative effect of sham acupuncture remains to be confirmed.

Our study was unique in that the included studies of acupuncture used the deep pricking method instead of the ordinary acupuncture method. The depth of the deep pricking method is deeper than that of ordinary acupuncture method. Further studies are needed to confirm whether the deep pricking method has a better curative effect on chronic constipation than ordinary acupuncture. In the present study, many studies conducted after 2012 were included and the studies using the same acupuncture points were included to ensure consistency. RCTs using consistent acupuncture points will yield more definitive results. However, the therapeutic effect of acupuncture in this study was based on the indirect curative effect of lactulose compared with placebo, and further studies are needed to investigate the direct effects of acupuncture and placebo.

A previous network meta-analysis of idiopathic constipation showed that the primary curative effect (> 3 CSBM(complete spontaneous bowel movement)per week or 1 CSBM greater than baseline per week) is similar between prucalopride, velusetrag, tegaserod, lubiprostone, elobixibat, bisacodyl, sodium picosulfate and linaclotide. As the secondary outcome, bisacodyl was found to be more efficacious than other drugs (including continuity or qualitative indicators) but was accompanied by side effects [56]. However, the previous study did not rank the side effects. In our study, five additional commonly used drugs (prucalopride, tegaserod, lubiprostone, bisacodyl, and linaclotide) were included and polyethylene glycol, lactulose, acupuncture and sham acupuncture were compared, as they are frequently used in our daily clinical practice. We analysed not only the curative efficacy but also side effects.

This study showed that the efficacy of polyethylene glycol is second only to acupuncture, and the side effects are minimal. The duration of the interventions ranged from 1 week to 24 weeks, covering long-term and short-term efficacy and side effects, and its effects were relatively positive. The acupuncture intervention time was relatively short in the majority of studies, so the comparison of long-term efficacy between acupuncture and polyethylene glycol requires further investigation. At the same time, this study did not distinguish between polyethylene glycol with or without electrolytes, but previous studies have shown that their efficacy is similar. [57]

This study also showed that the clinical effect of lactulose is acceptable, but the side effect profile is relatively unfavourable, including bloating and abdominal pain, but without serious adverse reactions. Because there was no direct comparison of side effects between lactulose and placebo, an indirect comparison to polyethylene glycol was conducted, which may have led to an overestimation of the real side effect profile of lactulose. Previous studies have shown that polyethylene glycol is superior to lactulose in the treatment of chronic constipation [58], which is consistent with the findings of the current study.

This study showed that the side effects of lubiprostone were more serious than those of linaclotide, prucalopride and bisacodyl, all of which were based on a direct comparison of side effects and were of clinical significance. At the same time, this study found that the curative effect of sham acupuncture was better than tegaserod, indicating that sham acupuncture may have some therapeutic effect, although it is based on an indirect comparison. In the past, many studies used sham acupuncture as a control group, but it is possible that the curative effect of acupuncture is underestimated because sham acupuncture has some curative effects. Related studies on the therapeutic effect of sham acupuncture have been conducted. [59]

This study also found that nearly all of the studies on acupuncture and chronic constipation used ST25 acupoints, while previous studies showed that ST25, ST36, L111, and BL25 may also have some beneficial effects on the motility of the distal colon. However, ST25 showed no effect on the distal colon of diarrhoea model rats [53]. The mechanism underlying the effects of different acupoints remains to be confirmed by further studies.

This study has several disadvantages. First, there were no direct comparisons between acupuncture and placebo and sham acupuncture and placebo. Second, the number of included studies for some drugs is small, and some study populations were regional, nearly 30% included articles were from China Some studies also lacked data on drug safety. All of these limitations lead to publication bias and may have impacted the results of our study. Third, the outcome of this study was the proportion of patients with overall symptom improvement. Fourth, the jaded score for risk assessment is relatively old. Lastly, this study did not include a comparison of short-term and long-term efficacy or consider time of disease onset or duration of disease. Such limitations lead to a certain gap in the clinical application of the findings of this study.

## Conclusions

In summary, this study found that acupuncture may be a good treatment option for chronic constipation with minimal side effects, but quality studies are still needed to support our findings. The curative effect of sham acupuncture should be further studied. Furthermore, polyethylene glycol is an acceptable treatment option with good curative effect and few side effects.

## Supporting information

S1 Table CFC:Chronic Functional Constipation; PRU:Prucalopride; TEG:Tegaserod; LUB:Lubiprostone; LIN:linaclotide; BIS:Bisacodyl; PEG:Polyethylene Glycol; PMF:Polyethylene glycol electrolyte balanced solution; PEG+E:polyethylene glycol+electrolytes; LAC:lactulose; ACU:acupuncture+electroacupuncture; SHAM ACU:sham acupuncture; int:international; CIC:chronic idiopathic constipation; STC:slow transit constipation; SF-36:Item Short Form Health Survey 36; PAC-SYM:Patient Assessment of Constipation symptom; PAC-QOL:Patient Assessment of Constipation-Quality of life; IVRS:interactive voice response system; BSFS: Bristol Stool Form Scale; HADS:Hospital Anxiety and Depression Scale; SBMS:spontaneous bowel movements; CCS:Cleveland Constipation Score; AGAMPSG:American Gastroenterological Association Medical Position Statement Guidelines; NA:Not available. (DOCX)

S2 Table The cumulative probability rankings of treatment effect of acupuncture on constipation. (TIFF)

S3 Table The cumulative probability rankings of side effect of drugs on constipation. (TIFF)

S1 Fig Brooks-Gelman-Rubin diagnostic plot of included studies. (TIFF)

S2 Fig Density plot of included studies. (TIF)

S3 Fig Node splitting plot of included studies. (TIFF)

S4 Fig The cumulative contribution plot of IBS-D treatment of Acupuncture compared with other drugs. PRU:Prucalopride; TEG:Tegaserod; LUB:Lubiprostone; LIN:linaclotide; BIS:Bisacodyl; PEG:Polyethylene Glycol; LAC:lactulose; ACU:acupuncture+electroacupuncture; SHAM ACU:sham acupuncture.
(TIF)

S5 Fig The heterogeneity analysis of included studies(1). A:Prucalopride; B:Tegaserod; C:Lubiprostone; D:linaclotide; E:Bisacodyl; F:Polyethylene Glycol; G:lactulose; H:acupuncture+electroacupuncture; I:sham acupuncture; J:Placebo.
(TIF)

S6 Fig The heterogeneity analysis of included studies(2). A:Prucalopride; B:Tegaserod; C:Lubiprostone; D:linaclotide; E:Bisacodyl; F:Polyethylene Glycol; G:lactulose; H:acupuncture+electroacupuncture; I:sham acupuncture; J:Placebo.
(TIFF)

S1 Checklist PRISMA 2009 checklist. (DOC)
